This article has been retracted.

# Super-resolution reconstruction of real infrared images acquired with unmanned aerial vehicle

**DOI:** 10.1371/journal.pone.0234775

**Published:** 2020-06-17

**Authors:** ZhengQiang Xiong, Qiuze Yu, Tao Sun, Wen Chen, Yuhao Wu, Jie Yin

**Affiliations:** 1 Electronic Information School, Wuhan University, Wuhan, China; 2 Shanghai Key Laboratory of Aerospace Intelligent Control Technology, Shanghai Institute of Spaceflight Control Technology, Shanghai, China; University College London, UNITED KINGDOM

## Abstract

Super-resolution (SR) technology provides a far promising computational imaging approach in obtaining a high-resolution (HR) image (or image sequences) from observed multiple low-resolution (LR) images by incorporating complementary information. In this paper, a three-stage SR method is proposed to generate a HR image from infrared (IR) LR Images acquired with Unmanned Aerial Vehicle (UAV). The proposed method integrates a high-level image capturing process and a low-level SR process. In this integrated process, we incorporate UAV path optimization, sub-pixel image registration, and sparseness constraint into a computational imaging framework of a region of interest (ROI). To refine ROI complementary feathers, we design an optimal flight control scheme to acquire adequate image sequences from multi-angles. In particular, a phase correlation approach achieving reliable sub-pixel image feature matching is adapted, on the basis of which an effective sparseness regularization model is built to enhance the fine structures of the IR image. Unlike most traditional multiple-frame SR algorithms that mainly focus on signal processing and achieve good performances when using standard test datasets, the performed experiments with real-life IR sequences indicate the three-stage SR method can also deal with practical LR IR image sequences collected by UAVs. The experimental results demonstrate that the proposed method is capable of generating HR images with good performance in terms of edge preservation and detail enhancement.

## 1 Introduction

Imaging devices have limited achievable resolution due to several theoretical and practical restrictions. Different theories reveal that an optical imaging system acts as a low-band pass filter, sparing the low spatial frequencies of an object’s spectrum but cutting off high frequency information [1]. Some of the high-spatial frequency signal information will be lost almost completely, due to the finite size of the lens apertures. Knowing how to obtain a high-resolution (HR) image is still an important and fundamental research topic.

Due to recent advances in communication, sensing, and battery technologies, UAVs have drawn much attention for both military and civilian applications. Thanks to their portability and maneuverability, UAVs are employed in numerous applications, including industrial monitoring, scientific data collection, and public safety (search and rescue) [2, 3]. Soon, autonomous aircraft equipped with various sensors will be routinely surveilling our cities, neighborhoods, and rural areas. In these applications, visual information is crucial to make decisions by a supervisor. Nonetheless, taking aerial images of a large field will consume a large amount of time. A possible method to reduce the time cost is to maximize the height, however, this will reduce the optical detail of image. These problems limit the extensive applications of UAVs, especially when obtaining HR and precision images of target objects. Therefore, a super-resolution (SR) computational imaging technique is necessary.

An important technical problem must, however, be addressed: How can we reconstruct HR image with real-time performance in the target reconnaissance mission? SR reconstruction aims to generate HR images via existing LR image or sequential samples. SR reconstruction has been widely used in microscopic imaging these years [4–6]. However, this problem remains to be challenging in the field of telemetry systems research, as it involves physical constraints due to the cameras themselves and constraints due to their operating environment, as well as other operational requirements.

Several quintessential methods, such as nonuniform interpolation approach [7–9], frequency domain approach [10–14], deterministic approach [15–19], stochastic approach [20–23] and ML-POCS hybrid reconstruction approach [24] have been developed for SR reconstruction. Although these methods can provide optimal or near-optimal images to increase the resolution, they cannot guarantee detail enhancement, i.e., geometric feature of detected target. Several problems need to be tackled to generate high-quality SR images from computational imaging:

1. High-Accuracy Image Registration Method: A critical step in SR is the accurate registration of the LR images because proper registration techniques can suppress large and complex geometric distortions.
2. Accurate Regression Model: because this model characterizes the imaging system, its accuracy can fully determine the precision of the system parameters derived from the imaging results. On this basis, the input images are estimated depending on these parameters.
3. Stable Solution of SR Reconstruction Algorithm: Generally, the SR image reconstruction approach is an ill-posed problem because of the insufficient number of LR images and the ill-conditioned blur operators. Consequently, different regularization terms incorporating prior information about IR imaging characteristics are designed, which acts a leading role in image quality.

We assume in conventional SR that either the estimated motion parameters by existing registration methods are error-free or the motion parameters are known as a priori knowledge [25, 26]. This assumption, however, is impractical in many applications, as most existing registration algorithms still experience various degrees of errors, and the motion parameters among the LR images are generally unknown. Due to the presence of aliasing in the captured LR images, most existing registration algorithms for aliased images still encounter sub-pixel errors.

Evgeniou [27] applied regularization to machine learning for the first time. After that different forms of regularization terms have been designed on the basis of certain requirements to solve the above ill-posed problem. Tikhonov regularization was employed by Hennings-Yeomans and Baker [28] because of the method’s mathematical simplicity. However, Tikhonov regularization belongs to a quadratic norm and unavoidably blurs image details. Ng et al. [29] and Chan et al. [30] utilized TV functions to characterize the HR images. Nevertheless, both of these approaches involve certain model parameters to be set by the users, which is a difficult task in general. Although deep learning technique has been gradually widely used in SR field in recent years [31–34], these algorithms generally achieve good performances only when using standard test datasets and need large amounts of training data to adjust the network parameters. In our work, a *l*_*p*_ norm-based regularization function is proposed against weak edge preservation of IR images, which fits the sparse characters of IR images and achieve fast-convergence performance.

Considering that the IR light has a longer wavelength than visible light, the IR cameras are able to detect targets beyond the visually distinguishable range. Besides, IR cameras provide excellent spatial correlation among neighborhood pixels. These characteristics make IR cameras widely popular when equipped by UAVs. For these reasons, we consider the reconstruction problem for IR cameras in this study. The aim of this study is to develop a UAV-equipped IR super-resolution reconstruction strategy to explicitly account reconstruction precision and efficiency. In this study, a UAV flight-path optimization algorithm and an edge-preserving sparse representation-based reconstruction method are proposed to solve the problem of multi-angle image acquirement and edge information retention. The specific contributions of this study are as follows:

1. An on-board IR image reconstruction framework is proposed to generate HR images that meet both real-time and precision requirements.
2. A UAV flight-path optimization method has been proposed, which provides optimal state parameters of UAVs for SR.
3. A sub-pixel image registration, which is absolutely necessary for eliminating pixel deviation, is developed in SR reconstruction process of image sequences, dramatically improving the accuracy of results.
4. A geometric shaping of the reconstructed image can be systematically performed with the designed sparseness constraint condition.

The rest of this paper is organized as follows. The problem formulation is presented in Section 2, where we make a further explanation for the problem to be solved through simple mathematical models. In Section 3, a three-stage SR method is proposed and the workflow of our method is presented from the overall aspects and the detail respectively. Section 4 shows the simulation and experimental results to demonstrate the performance of the proposed method. Section 5 draws the conclusion of our study.

## 2 Problem formulation

LR IR image sequences from multiple views are fused to generate a HR IR image in this study. Traditional multiple-frame SR algorithms usually focus on signal processing and can achieve good performances when using standard test datasets. However, practical LR IR image sequences collected by UAVs can hardly provide enough complementary information without a flight control strategy. In our work, a high-level IR image capturing method and a low-level SR reconstruction algorithm are integrated to produce HR IR image.

Let g_k_ be k LR frames acquired from the original scene. The SR reconstruction problem estimates the HR image of the original scene, which is denoted as the HR image f of size F * F. The LR frames are linked with the HR image through a series of degradations. The formulation of the LR images in the vector-matrix notation is described as:

$$g_{k}=DV_{k}W_{k}f+n_{k}$$ (1)

where V_k_ denotes the blur matrix, W_k_ represents the warp matrix, n_k_ is the additive noise present in each image process. The decimation matrix D = SU simulates the behavior of digital sensors by first performing convolution with the sensor S and the sampling operator U. The sensitivity of the sensor is highest in the middle and decreases towards its borders with a Gaussian- like decay. Furthermore, the down-sampling factor (or SR upscale factor, depending on the point of view), denoted by ε, is assumed to be the same along both x and y directions. It should be noted that ε is a user-defined parameter. The sub-pixel accuracy in g_k_ has been proven necessary for SR to work. Standard image registration techniques can hardly achieve this goal, and they leave a small misalignment behind. Therefore, we will assume that complex geometric transforms are removed in the prepossessing step, and W_k_ is reduced to a small translation *H*_*k*_. Consequently, the acquisition model becomes

$$g_{k}=SUH_{k}f+n_{k}$$ (2)

Then, the SR problem adopts the following form: provided LR images g_k_, we want to estimate the HR image f for the given S. In improving the quality of SR results, sufficient observation sequences are indispensable to provide complementary information in space. To achieve this, a three-stage SR method is proposed to integrate a high-level image capturing and a low-level SR process, in which we incorporate UAV path optimization, sub-pixel image registration, and sparseness constraint into a computational imaging framework of a region of interest (ROI).

## 3 Three-stage sr method

Three-stage SR method is proposed in this work to deal with problems involving on-board image reconstruction for small-target detection. The operational workflow of this algorithm is presented in Fig 1.

**Fig 1:** Workflow of the edge-preserving and detail-enhancement SR algorithm.

As shown in Fig 1, our algorithm has three key steps: UAV flight control, image registration and sparseness constraint. Sufficient observation samples are required to improve SR accuracy. Given that the changes in flying altitude directly lead to inconsistent observation resolutions, a flight optimization strategy should be developed to get adequate image sequences from multiple views, while keeping a consistent resolution in general. Then, a sub-pixel registration method is proposed to eliminate the pixel deviation caused by the UAV motion. Subsequently, in ensuring that the HR images preserve edge information, a sparseness regularization constraint scheme is used to recover the missing high-frequency information on the basis of Stage-2.

### 3.1 Consistent resolution and multi-angle observation-based flight control

In this work, the UAV equipped with an IR camera is designed to run in a “stare-step-stare” manner, as shown in Fig 2. Once a suspected small target appears in the field of view, the UAV is schemed to hover and “stare” at the ROI for a certain period. In this process, the UAV generally stays in a stable state, guaranteeing that IR image sequences of ROI are acquired. Meanwhile, the UAV jitters slightly while hovering, and produces complementary information between pixels is produced. The time of “stare” can be set according to the frame rate of the IR camera, then the UAV switches into “step” mode until it finds another interested target. The resolution of the acquired snapshot is decided on the basis of object distance and shooting angle. Thus flight parameters including velocity, pose, and position must be adjustable to guarantee the effective resolution of IR images.

**Fig 2:** UAV flight control.

Geometric features, including texture, shape, and spatial relations of sampled images, provide important structure information of the original images. However, these high-dimensional features can hardly be exacted simultaneously via single sampling, due to imperfect lighting condition and potential obstruction. Multi-angle technology, can potentially be used to solve the incomplete observation problem. In particular, a UAV can be scheduled to a predesigned position to view the path planning, and subsequently helps to collect specific details. Additionally, image resolution consistency is another concern in this study. For simplicity’s sake, the image resolution with consistency is defined as the Effective Resolution (ER) as elaborated in Fig 3a. Images with higher ER values provides much more geometrics characteristics information. Furthermore, extracting useful information from low ER value images is arduous. In order to improve observation efficiency and data precision, ER consistency is required, as it essentially brings constraints on the pose of an on-board camera.

**Fig 3:** Optimal path planning for consistent resolution and multi-angle observations.

A UAV is generally powered by batteries or gasoline. Compared with gasoline-driven UAVs, power- supplied UAVs are more advanced in many aspects. Power-supplied UAVs have the advantages of better flexibility because of their lightweight airframe. More importantly, they tend to be more suitable for flying in urban environments, as batteries are known to have a stable performance, and thus, safety can be ensured. For these reasons, we also consider the path-planning problem for power-supplied UAVs in this work.

Considering the aerodynamics of a UAV, the path-planning problem can be formulated as follows:

$$\underset{{}_{u\left(t\right)\in \Omega }}{\text{min}}J\left(u\right)=\varphi \left(X\left(t\right)\right)+\int_{t_{0}}^{t_{f}}L\left(X,U\right)dt$$ (3)

$$s.t.\dot{X}\left(t\right)=f\left(x,U,t\right),x\left(t_{0}\right)=X_{0},\Psi \left[x\left(t_{0}\right)\right]=0$$

where Ψ(·) is the constraint condition, ϕ(·) denotes the end term, **X** represents the UAV state, and L is the optimization goal.

The automatic control and dynamic optimization (**ACADO**) tool is employed to obtain the optimized solution for the above problem. Given that the dynamics of a UAV is a coupling process involving several variables, it is difficult to be solved by analytical methods. The ACADO toolkit is a software environment and an algorithmic collection for automatic control and dynamic optimization. **ACADO** provides a general framework in using a great variety of algorithms for direct optimal control, including model predictive control, state and parameter estimation and robust optimization. Considering these advantages, **ACADO** is used to solve the optimization problem in this work.

### 3.2 Robust phase correlation registration algorithm

The motion parameters among the LR IR images are generally unknown in advance, hence a critical step in SR is the accurate registration of the LR images. Proper registration techniques can suppress large and complex geometric distortions [24]. Sub-pixel accuracy is necessary for SR to work. However, standard image registration techniques can hardly achieve this goal and they leave a small misalignment behind. In our work, the geometric transforms are removed in the preprocessing steps, including UAV flight control and image registration, with sub-pixel accuracy.

Let *g* (*x*, *y*) and *h* (*x*, *y*) be two 2D functions representing two images related by a simple translational shift *a* in horizontal and *b* in vertical directions. According to the Fourier shift property

$$\hat{h}\left(\text{x},y\right)=\hat{g}\left(\text{x},\text{y}\right)exp\left\{-i\left(a\text{x}+b\text{y}\right)\right\}$$ (4)

Hence, the normalized cross power spectrum can be described as follows:

$$Q\left(u,v\right)=\frac{G\left(u,v\right)H{\left(u,v\right)}^{⋆}}{\left|G\left(u,v\right)H{\left(u,v\right)}^{⋆}\right|}=exp\left\{-i\left(au+bv\right)\right\}$$ (5)

where *G*(*u*, *v*) and *H*(*u*, *v*) represent the Fourier Transform of g(x, y) and h(x, y)respectively, * indicates the complex conjugate.

The inversed Fourier Transform (*IFT*) of *Q*(*u*, *v*) is a delta function, as shown in Eq (6), when *G*(*u*, *v*) and *H*(*u*, *v*) are continuous functions,

q(x,y)=δ(x−a,y−b) (6)

in which the function peak identifies the magnitude of the shift.

Given the raster data of images, *q*(*u*, *v*) presents a delta-like function, and subsequently, the translation estimation between the two related images represented by functions $\hat{g}\left(u,v\right)$ and $\hat{h}\left(u,v\right)$ can only be performed at integer (pixel) accuracy, even though the true shift a and b can be real numbers with decimal parts (or sub-pixels).

In order to realize the translation estimation at sub-pixel accuracy based on Eq (6), over-sampling is generally employed to generate sub-pixel level images before the FT phase. However, the computing load will be increased dramatically. To reduce calculation burden, we consider direct solutions according to the phase correlation matrix defined in Eq (5). As the magnitude of Q(u, v) is normalized to 1, the only variable in Eq (5) becomes the phase shift defined by au + bv. Consequently, the non-integer translation estimation at sub-pixel accuracy can be achieved without applying IFT if *a* and *b* can be accurately figured out. Such a frequency domain approach has been proven to be more effective in achieving accuracy and speed than that based on the delta function of Eq (6).

Recognizing that Q(u, v) is in fact equivalent to a rank one complex matrix, then Q(u, v) can be decomposed into the two vectors of u and v,

Q(u,v)=exp{−iau}exp{−ibv} (7)

Given that

$$q_{a}\left(u\right)=exp\left\{-iau\right\},q_{b}\left(v\right)=exp\left\{+ibv\right\}$$ (8)

then

$$Q\left(u,v\right)=q_{a}\left(u\right)q_{b}{\left(v\right)}^{*}$$ (9)

Considering that singular value decomposition (SVD) [35] is advanced in data simplification as well as noise elimination, it is used to find the dominant rank-one subspace of *Q*. As a result, linear phase coefficients can be identified independently in the left and right dominant singular vectors based on Eq (9). This approach implements a 2D phase unwrapping with two independent 1D phase unwrapping based on the left and right dominant singular vectors. The Least Square Fit (LSF) to the unwrapped phase component of the dominant singular vectors provides estimates of the vertical and horizontal shift for non-integer translational motion over a large range. However, the problem of slow computation speed hinders its practical applications as the SVD is in complex matrix operations.

The data of the phase correlation matrix *Q* (*u*, *v*) defined by Eq (5) can be understood in simple geometry. The phase shift angle in Eq (5) is

c=au+bv (10)

This equation is simply a 2D plane in *u − v* coordinates defined by the coefficients *a* and *b*. The image shift magnitudes *a* and *b* can be solved by the rank-one approximation of the phase correlation matrix Q(u, v). However, the phase shift angle *c* is 2*π-*wrapped in the direction defined by *a* and *b*. The 2D unwrapping can be performed by two separate and consecutive 1D unwrapping in direction of *u* and *v*.

A direct 2D LSF based on Eq (10) can avoid the complex matrix operations of SVD. However, it has been proved that 2D unwrapping on the phase angle data in the Q(u, v) is often unreliable and resulting in failure of finding a and b correctly which is mainly caused by noisier data of Q(u, v). Although the 2D fitting method is much faster than the SVD one, it suffered from large magnitude shifts and rotation.

To overcome the drawback of 2D fitting method, data noise was reduced before unwrapping. Here, a phase fringe filtering technique is designed as below:

***step*1**. Denote θ(u, v) as the phase angle at position u, v in the phase correlation matrix Q(u, v).
***step2***. The sinθ and cosθ are continuous functions of θ(u, v), a smoothing filter can therefore be applied to these functions.
***step 3***. Derive the filtered phase angle $\bar{\theta \left(u,v\right)}$ from the smoothing-filtered sinθ and cosθ:

$$tan\bar{\theta }=\frac{\bar{sin\theta }}{\bar{cos\theta }}$$ (11)

It should be noted that the window size of the smoothing filter must be small in comparison to the half wavelength of sinθ and cosθ.

### 3.3 Sparse representation-based super-resolution reconstruction method

IR images generally suffer from a relatively low radiation intensity, resulting in crucial edge information loss, which is adverse to small targets detection. Our work is focused on recovering high-frequency information through LR IR images without too much time complexity.

Inspired by the approach taken by Sroubek et al. [24] in which a regularized energy function was built and minimized with respect to the original images and blur domains, we extend the framework to develop a phase correlation-based SR reconstruction algorithm. Fig 4 shows the observation model of the proposed method. Different from the previous method, rectified images produced by the phase correlation algorithm act as the initial value of the iteration (Fig 5). Moreover, we also build a sparse representation function to extrapolate the optimal reconstruction parameters.

**Fig 4:** Thermal IR imaging model.

**Fig 5:** Super-resolution reconstruction workflow.

The image degradation process can be modeled as:

$$y_{k}=DHF_{x}+N,k=1,\cdots ,K,N\sim N\left(0,W^{-1}\right)$$ (12)

where *D* denotes downsampling, *H* denotes the blur process, *F*_*k*_ represents the warp matrix, *N* is the additive noise. The super-resolution reconstruction can be regarded a reverse operation of Eq (12), which is essentially an ill-posed problem if no priori information exists. However, the SR can be converted into an optimization problem of the minimized cost function with the regularization method. On the basis of the image degradation process, the SR solution is formulated as:

$$\hat{X}=argmin\sum_{k=1}^{K}{\left\|DHF_{k}X-y_{k}\right\|}_{2}+\lambda_{1}f_{BTV}\left(X\right)+\lambda_{2}f_{\delta }\left(X\right)$$ (13)

where $\hat{X}$ represents the HR image to be estimated, ∥·∥_2_ is the *l*_2_-norm, *f*(*X*) denotes the regularization term, and λ is the regularization parameter.

According to the amplification factor of SR, the iterative initial value *X*0 is first generated by averaging the upsampling LR IR image sequences. The BTV regularization item is employed as a smoothness constraint in our method. Numerous criterions for regularization are designed, typical of which include Tikhonov and TV. However, the BTV item not only has good robustness to noise, but also improves smoothness while alleviating effectively the ringing artifacts generally resulted from deconvolution algorithm. These characteristics enable make BTV to become more suitable for remote sensing images. The BTV term takes the following form:

$$f_{BTV}\left(X\right)=\sum_{l=-P}^{P}\sum_{m=-P}^{P}\omega^{\left|m\right|+\left|l\right|}{\left\|X-S_{x}^{l}S_{y}^{m}X\right\|}_{1}$$ (14)

where $S_{x}^{l}$ and $S_{y}^{m}$ are the translation operators in the horizontal and vertical directions, ***P*** represents the moving range (***P*** > 1), and *ω* is the weight coefficient (0<*ω*< 1).

Besides the smoothness constraint, a sparseness constraint formula is also designed for the first time as part of our algorithm. It has been demonstrated that the main information and the internal structure of images can be mapped (captured) by a few coefficient via sparse representation. Moreover, this strategy has been proven to have stronger adaptability and better robustness to noise and errors compared with the previous method.

An objective function with *l*_*p*_-norm (0 *< p <* 1) regularization item is built to obtain a stable sparse solution. Although regularization with the *l*_1_-norm is a convex optimization problem, and a fast method can be used to solve it, the sparseness and robustness of the solution are inferior. Meanwhile, the problem with *l*_0_-norm belongs to combinatorial optimization, which is too complicated to be resolved and disadvantaged in practical applications. Thus, *l*_*p*_-norm (0 *< p <* 1), characterized in strong noise resistance and loose reconstruction condition, is employed to figure out sparse solution.

By submitting Eqs (14) to (13) and taking ∥·∥_*p*_ as *l*_*p*_-*norm*, we obtain

$$\hat{X}=argmin\frac{1}{2}\sum_{k=1}^{K}{\left\|DHF_{k}X-y_{k}\right\|}_{2}+\lambda_{1}{\left\|BTV\left(X\right)\right\|}_{1}+\lambda_{2}{\left\|X\right\|}_{p}$$ (15)

A continuously differentiable function is defined to approximate *l*_0_-norm. The same definition is also followed in this work, that is,

$$f_{\delta }\left(x\right)=tan\frac{\pi x^{2}}{4\left(\delta^{2}+x^{2}\right)}$$ (16)

and then conclude that

$$\underset{\delta \to 0}{\text{lim}}f_{\delta }\left(x\right)=\{\begin{array}{ll} 1\;x\neq 0 & \\ 0\;x=0 & \end{array}$$ (17)

Afterwards, the *l*_0_-norm approximation takes the form,

$${\left\|X\right\|}_{0}\approx \sum_{i-1}^{N}f_{\delta }\left(x_{i}\right)={\left\|X\right\|}_{p}$$ (18)

As demonstrated in Fig 6, results of the numerical calculation show that the above formula entails a sparsity of IR images with fast convergence. Thus, the formula is feasible for approximating the *l*_0_-norm for edge restriction.

**Fig 6:** Diagram of sparse function designed in our work.

Compared with conventional search algorithms, the steepest descent method has the advantages of low space complexity and quick convergence speed even when the results are far from the local extremums. Thus, it is used to determine the optimal parameters of the construction.

## 4 Experiments and validation

The effectiveness and robustness of the SR method is verified by using an eight-rotor UAV equipped with HSN120A IR camera for the physical experiments, as shown in Fig 7. The UAV follows a predefined path for energy conservation in a “stare-step-stare” mode to sample the observation site. The experimental results are shown in Figs 8–10. The enlarged parts of the SR images are also displayed in Figs 8–10. The demonstrations indicate that the selected part has several dominant edges of different targets. Meanwhile, it also shows that the SR image with well-preserved edges and less overshot effects compared with LR images.

**Fig 7:** Experimental scene: An eight-rotor UAV equipped with HSN120A IR camera, with experiment conducted around Zhuoer Gymnasium in Wuhan University.

**Fig 8:** Experimental result of Target 1.

**Fig 9:** Experimental result of Target 2.

**Fig 10:** Experimental result of Target 3.

Fig 8 presents 100 LR aerial IR images and the × 4 upscale SR result. These IR images were obtained from the ASL datasets of ETH Zurich (https://projects.asl.ethz.ch/datasets). They were recorded using a handheld FLIR Tau 320 thermal IR camera with a resolution of 324 × 256 pixels which were simulated to be captured by UAV under the ideal condition. Even so, the geometric features still degraded in raw images due to low resolution which makes the target indecipherable in vision. By super-resolution reconstruction, the edge and texture features of tile on roof has been remarkably enhanced on SR result. Also, the architectural feature of stairs on ground is much more notable compared with that in LR images since three flights of steps are clearly visible. It indicates that higher spatial frequency components have been recovered from the low resolution images without introducing ringing artifacts, which will bring much convenience to target identification.

Fig 9 shows 100 LR real IR images acquired with UAV fight control and the corresponding × 4 upscale SR result. This group of image sequences were acquired by an eight-rotor UAV equipped with HSN120A IR camera, whose original resolution is 704 × 576 pixels. The SR result shows that the spatial resolution has been effectively improved with much finer structures and sharp edge. It can be seen that the local geometric distortions (A straight line becomes a broken line) are rectified and detail information of windows as well as handrail is highlighted. It proves that our method is able to remove stripe noises while preserving the original image details as much as possible so that the original features of various targets could be obtained better through IR imaging.

Furthermore, a reconstruction experiment is conducted especially for text objects to demonstrate the validity and practicability of the proposed model and algorithm, as shown in Fig 10. These LR IR images were collected in the same manner as that for Fig 9 and cut out the part of the text target. In the original LR images, the string “school” is hard to recognize owing to the discontinuous edges caused by low resolution configuration of the IR cameras. However, the high-spatial frequency information is retrieved via complementary information from sequential images, and the mended broken characters have smooth edges and a complete structure, which meet the need of the next target feature extraction.

We also compare the performance of three different state-of-the-art SR methods to evaluate the performance of the proposed SR reconstruction algorithm. The results from S1 Dataset in Fig 11 shows that our method can restore the textural features of three flights of the steps. Although the image size is increased, the edge and detail information of high frequency are still missed by Bicubic, POCS and TV. As shown by S2 Dataset, the geometric distortions are rectified to some extent by POCS and TV, but the collected images suffered from lower contrast and lower detailed nature compared with that of our method. S3 Dataset does, however, indicate our method is advanced in continuity of edges and sharpness of the images. Compared with the other three SR methods, our method performs better in terms of high-spatial frequency information recovery and edge preservation against IR images of different targets. The overall finding provides the basis of target reconnaissance and detection of UAVs.

**Fig 11:** Performance comparison of different super-resolution results.

In order to measure the performance of the proposed method quantitatively, an energy of gradient (*EOG*) index is introduced into each methods. It is formulated as

$$EOG=\sum_{1}^{Y}\sum_{1}^{X}(|f(x+1,y)-f(x,y){|}^{2}+|f(x,y+1)-f(x,y){|}^{2})$$ (19)

where *g*(*x*, *y*) is the gray value of pixel (*x*, *y*).

EOG can measure the image sharpness to some extent and express the high-frequency components of an image. In the experiments with the three sets of real IR images, the performance of the proposed method is compared with that of three conventional methods. The EOG indexes of the original LR IR images and the corresponding results of each SR methods are presented in Fig 12. It is noted that the results of the proposed method are better than the original LR IR images, as well as the results of the other three methods.

**Fig 12:** Quantitative comparison of different methods.

## 5 Conclusions

A sparse representation based super-resolution framework for on-board high resolution IR imaging is proposed in this study to integrate a high-level image capturing and a low-level super-resolution process. A path-optimal UAV flight control method is designed to acquire sufficient multi-angle image sequences, serving for small targets detection. Subsequently, a sub-pixel image registration algorithm is developed to eliminate pixel deviation. In particular, a sparseness constraint mechanism is established in accordance with the textural features of the images. The results demonstrate that the algorithm is capable of generating HR images with good performance in terms of edge preservation and detail enhancement. To our knowledge, our proposed method is one of the first methods used for simultaneous UAV control and resolution enhancement.

Although the proposed method has achieved satisfactory results, this work is just the beginning to implement this automated approach in IR image SR reconstruction. In this work, the UAV is assumed to achieve steady attitude by proposed optimal control methods. However, external disturbances (e.g., wind field) would inevitably induce displacement, jitter and blurring of images. In further works, we will develop a motion deblurring algorithm incorporated into our research, and we are also interested in evaluating the effect of AOV (angle of view) on SR results.

## Supporting information

S1 Dataset (ZIP)

S2 Dataset (ZIP)

S3 Dataset (ZIP)

S1 File (DOC)
